This article has been retracted.

# Chinese Herbal Medicine Suppresses Invasion-Promoting Capacity of Cancer-Associated Fibroblasts in Pancreatic Cancer

**DOI:** 10.1371/journal.pone.0096177

**Published:** 2014-04-29

**Authors:** Lianyu Chen, Chao Qu, Hao Chen, Litao Xu, Qi Qi, Jianmin Luo, Kun Wang, Zhiqiang Meng, Zhen Chen, Peng Wang, Luming Liu

**Affiliations:** 1 Department of Integrative Oncology, Fudan University Shanghai Cancer Center, Shanghai, China; 2 Department of Oncology, Shanghai medical college, Fudan University, Shanghai, China; University of Bergen, Norway

## Abstract

Pancreatic cancer remains one of the leading causes of cancer-related deaths, due to aggressive growth, high metastatic rates during the early stage and the lack of an effective therapeutic approach. We previously showed that Qingyihuaji (QYHJ), a seven-herb Chinese medicine formula, exhibited significant anti-cancer effects in pancreatic cancer, associated with modifications in the tumor microenvironment, particularly the inhibition of cancer-associated fibroblast (CAF) activation. In the present study, we generated CAF and paired normal fibroblast (NF) cultures from resected human pancreatic cancer tissues. We observed that CAFs exhibited an enhanced capacity for inducing pancreatic cancer cell migration and invasion compared with NFs, while QYHJ-treated CAFs exhibited decreased migration and invasion-promoting capacities in vitro. The results of further analyses indicated that compared with NFs, CAFs exhibit increased CXCL1, 2 and 8 expression, contributing to the enhanced invasion-promoting capacities of these cells, while QYHJ treatment significantly suppressed CAF proliferation activities and the production of CAF-derived CXCL1, 2 and 8. These in vitro observations were confirmed in mice models of human pancreatic cancer. Taken together, these results suggested that suppressing the tumor-promoting capacity of CAFs through Chinese herbal medicine attenuates pancreatic cancer cell invasion.

## Introduction

Due to aggressive growth and a high metastatic rate during the early stage, pancreatic cancer remains a highly lethal malignant disease [1], and only approximately 10–20% of pancreatic cancer is resectable at the time of diagnosis [2]. Gemcitabine has been the standard treatment for advanced pancreatic cancer; however, the median survival is 5–6 months, with the frequent development of chemo-resistance during the treatment [3]. Thus, pancreatic cancer remains a dreadful disease, and there is an urgent need of further studies to reveal the molecular mechanisms of tumor invasion and metastasis to develop an effective therapeutic approach to prevent and/or treat of pancreatic cancer.

Cancer associated fibroblasts (CAFs), predominant components of the tumor stroma, have been extracted from several invasive human carcinomas, including pancreatic cancer [4], [5], [6]. Pancreatic ductal adenocarcinoma is characterized by an extensive stromal response called desmoplasia [7]. Within the tumor stroma, CAFs are the primary cell type, which play an important role in tumor progression [5]. CAFs secrete multiple factors, including CXC, CC chemokines, and other inflammatory mediators, that promote the proliferation, invasion, and metastasis of cancer cells. Moreover, accumulating evidence has demonstrated that CAFs play a key role in the acquisition of drug resistance in tumor therapy [8], which negatively impacts clinical outcomes [9], [10]. Therefore, inhibiting the activation of CAFs might represent a potential therapeutic approach for pancreatic cancer treatment.

QYHJ, a seven-herb Chinese medicinal formula used for treating pancreatic cancer in China, inhibits both tumor growth and metastasis in nude mice models of pancreatic cancer [11], [12], [13]. In addition, the combined use of QYHJ with conventional Western medicine prolongs survival time in patients with liver metastases from pancreatic cancer [14]. However, the underlying molecular mechanism remains unclear.

Here, we demonstrated that CAFs exhibited an enhanced capacity for inducing pancreatic cancer cell migration and invasion compared with NFs, while QYHJ-treated CAFs exhibited decreased migration- and invasion-promoting capacities in vitro. In addition, we showed that compared with NFs, CAFs express high levels of CXCL1, 2 and 8, contributing to the enhanced invasion-promoting capacity of these cells. Thus, QYHJ treatment could suppress the proliferation activities and CXCL1, 2 and 8 expression levels in CAFs. Taken together, these results suggest that suppressing the tumor-promoting capacity of CAFs with Chinese herbal medicine attenuates pancreatic cancer cell invasion.

## Materials and Methods

### Ethics Statement

All animal experiments were conducted in accordance with the guidelines of the National Institutes of Health for the Care and Use of Laboratory Animals. The study protocol was also approved through the Committee on the Use of Live Animals in Teaching and Research, Fudan University, Shanghai. At the end of the study, all animals were decapitated through spinal cord separation at the nuchae to minimize suffering. The fibroblasts were isolated from resected tissues of two patients with pancreatic ductal adenocarcinomas (PDAC). Before sample collection, written informed consent was obtained from each patient in accordance with institutional guidelines, and the study was approved through the committees for the ethical review of research at the Fudan University Shanghai Cancer Center.

### Cell Lines and Mice

The human pancreatic cancer cell line Capan1 and BxPC3 were obtained from the American Type Culture Collection, and cultured in Dulbecco's modified Eagle medium (DMEM; Gibco, Carlsbad, CA) supplemented with 10% fetal bovine serum (FBS; Gibco, Carlsbad, CA) at 37 °C with 5% CO_2_. The morphology of the Capan1 cell line was regularly assessed, and the cells were tested for the absence of mycoplasma contamination (MycoAlert, Lonza, Rockland, ME, USA). The Capan1 and BxPC3 cell lines at the 30∼40 passages were used in our study.

Female BALB/c-nu/nu nude mice aged 4–6 weeks were obtained from the Shanghai Institute of Materia Medica, Chinese Academy of Sciences (Shanghai, China), housed in laminar flow cabinets under specific pathogen-free conditions and provided food and water *ad libitum*.

### Isolation of CAFs and paired NFs

Stromal fibrolasts were isolated as previously described [15]. Briefly, surgically resected pancreatic cancer tissues were obtained from two patients with pancreatic ductal adenocarcinoma. Written informed consent was obtained before tissue collection. The fresh pancreas tumor tissue and adjacent normal tissue (at least 2 cm from the outer tumor margin) were minced into 1–3 mm^3^ fragments and digested with 0.25% trypsin at 37°C for 30 min. The resulting fragments were centrifuged at 600 xg for 5 min and washed once with DMEM containing 10% fetal bovine serum. The tissue fragments were subsequently plated and incubated at 37°C. The culture medium was changed twice a week for 3–4 weeks. Under these conditions, fibroblasts were explanted from tissue fragments while other cells were mostly retained in the tissue. Fibroblasts formed multi-layer colonies spreading on the culture dish. After 3–4 weeks cultured cells were roughly trypsinized and re-plated into T25 culture flasks (passage one). The fibroblasts were then sub-cultured for another 2–3 passages until the cultures were free of contamination of epithelial cells and subsequently maintained in DMEM supplemented with 10% fetal bovine serum, 2% penicillin and streptomycin (Invitrogen, Carlsbad, CA, USA). The cells were grown at 37°C in a humidified atmosphere containing 5% CO_2_.NF and CAF strains were used at the 4–5 passages.

### Immunohistochemistry and immunofluorescence

Immunohistochemistry (IHC) was performed as previously described [16]. Briefly, the tumor tissue samples were fixed in 10% formalin and embedded in paraffin wax. Unstained 3-µm sections were subsequently cut from the paraffin blocks for IHC analysis. The sections were stained with the following antibodies: rabbit anti-vimentin (1∶200), rabbit anti-α-SMA (1∶100), rabbit anti-CXCL1 (1∶100), rabbit anti-CXCL2 (1∶200), and rabbit anti-CXCL8 (1∶25) at 4°C overnight. The sections were incubated with secondary antibodies, and the avidin-biotin peroxidase complex was used according to the manufacturer's instructions (Vector Laboratories, CA, USA). An immunoglobulin-negative control was used to rule out non-specific binding. Two independent investigators and one pathologist, all of whom were blinded to the model/treatment type for the series of specimens, performed all procedures. To quantitatively evaluate the CAF-induced proliferative activity in each group, we calculated the ratio of the area positive for vimentin and α-SMA staining to the total area in histological sections from ten fields under light microscopy (200×) [11].

For immunofluorescence staining, the cells were fixed with 4% paraformaldehyde and incubated with anti-Pan-CK (1∶100), anti-α-SMA (1∶100), anti-vimentin (1∶100), anti-E-cadherin (1∶100), anti-CD31(1∶200) and anti-D2-40 (1∶100) at 4°C overnight. The cells were subsequently incubated with fluorescence-conjugated secondary antibody for 1 h. After washing, the cells were mounted with mounting medium containing DAPI (Vector Laboratories). A negative control, in which the primary antibody was omitted, was used to test for antibody specificity. The images were captured using a confocal Leica fluorescence microscope.

### Drugs and Reagents

QYHJ, a seven-herb Chinese medicinal formula, comprised *Scutellria barbata* (Ban zhi lian), *Heydyotis diffusa* (Bai hua she she cao), *Amorphophallus kiusianus* (She liu gu), *Coix lacryma-jobi* (Yi ren), *Gynostemma pentaphyllum* (Jiao gu lan), *Ganoderma luncidum* (Ling zhi) and *Amomum cardamomum* (Bai dou kou), was prepared as previously decribed [11], [12], [13]. Briefly, QYHJ powder was obtained from Jiang-yin Tianjiang Pharmaceutical Co, Ltd. To ensure standardization and maintain the interbatch reliability of QYHJ, a high performance liquid chromatography (HPLC) chromatographic fingerprint was developed for quality control. The fingerprint chromatograms of QYHJ formula are shown in our previous report [17]. The final decoction of QYHJ was prepared after dissolving the herbal powder in distilled water to the required concentration. The daily dosage for rabbit and nude mice was 15 g/kg and 18 g/kg, respectively, calculated according to the following human-rabbit or human-mouse transfer formula: Db  =  Da × (Rb/Ra) × (Wb/Wa)2/3, where D, R, and W represent dosage, shape coefficient, and body weight, respectively, and a and b represent human and mouse or rabbit, respectively. Human recombinant CXCL1, 2, and 8 were obtained from PeproTech (Rocky Hill, NJ, USA). The anti-CXCR1 blocking antibody was obtained from R&D Systems (Minneapolis, MN, USA). The CXCR2 inhibitor SB 225002 was obtained from Enzo Life Sciences, Inc. (Farmingdale, NY, USA). The following antibodies were used: anti-E-cadherin, anti-Vimentin, anti-α-SMA, anti-CXCL8, anti-CXCL1 (all from Epitomics, Burlingame, CA, USA), anti-Pan Cytokeratin (AE1/AE3) (Pan-CK; Ascend Biotechnology, Guangzhou, China), and anti-CXCL2 (Bioss, Beijing, China).

### Preparation of QYHJ-Containing Serum

The QYHJ-Containing Serum was prepared as previously described [18]. Briefly, 20 female rabbits, weighing 1800±2200 g, were randomly divided into two groups: the QYHJ-Containing Serum group and the vehicle control group. The QYHJ-Containing Serum group was gavaged with intragastric QYHJ once a day for 7 consecutive days (12.5 g/kg body weight/time), and the vehicle control group was gavaged with intragastric deionized water. Blood was collected from the carotid artery within 2 h after the last administration and incubated at room temperature for 2 h. The serum from the whole blood was centrifuged (4,000 r/min for 10 min) and inactivated in a 56°C water bath for 30 min. The serum was stored at −80°C, and repeated freezing and thawing were avoided.

### Migration and invasion assay

Cell migration and invasion were determined using transwell cell migration plates (Corning, NY, USA) and Matrigel invasion chambers (Matrigel-coated membrane, BD Biosciences, San Jose, CA, USA) as previously described [19]. Briefly, the cells (1.0×10^4^) were seeded in serum-free medium into the upper chamber and allowed to invade toward 10% FCS in the lower chamber as a chemoattractant. After 12 h (for migration assays without matrigel coating) or 48 h (for invasion assays with matrigel coating), the cells that had invaded through the membrane and adhered to the underside of the membrane were counted as previously described [16].

### Western Blot Analysis

Total protein was extracted from the cultured cells, and quantitated using the bicinchoninic acid assay kit (Pierce, Rockford, IL, USA). Western blotting was performed according to our previous report [16]. Equal amounts of protein from different samples were separated through 10% SDS-polyacrylate gel electrophoresis and transferred to a polyvinylidene fluoride membrane. Blocking buffer, containing 5% non-fat milk, was used to block and incubate the membranes with primary antibodies. The expression of the target proteins was examined using an enhance chemiluminescence (ECL) kit (Amersham Pharmacia Biotech, Uppsala, Sweden), and the quantitative analysis was performed using ImageJ software.

### RNA isolation and real-time PCR

Total RNA was isolated from the cells using TRIzol Reagent (Invitrogen, San Diego, CA, USA), and reverse transcription PCR (RT-PCR) was performed according to the manufacturer's instructions (TakaRa). Quantitative real-time PCR measurements were performed using SYBR green I (Roche Diagnostics, Branchburg, NJ, USA). The primer sequences for CXCL1, 2, and 8 are listed in Table 1. GAPDH was used as an internal control. All experiments were performed in triplicate and repeated twice.

**Table 1:** Primers and annealing temperatures used for RT-PCR.

Gene	Primer sequence		Product size (bp)	Annealing (°C)
CXCL1	F	5′-TGAAGGCAGGGGAATGTATGTG-3′	226	60
	R	5′-AGCCCCTTTGTTCTAAGCCAGA -3′		
CXCL2	F	5′-AGATCAATGTGACGGCAGGGA-3′	235	60
	R	5′-CTCTCTGCTCTAACACAGAGGGAA-3′		
CXCL8	F	5′-AAGCCACCGGAGCACTCCATA-3′	170	60
	R	5′-CGGCCAGCTTGGAAGTCATGT-3′		
GAPDH	F	5′-GGGAGCCAAAAGGGTCATCATCTC -3′	353	60
	R	5′-CCATGCCAGTGAGCTTCCCGTTC -3′		

### Conditioned medium (CM) preparation

CM from CAFs and NFs was obtained as previously described, with slight modifications [20]. Briefly, the cells were maintained in DMEM at 37°C for 48 h. The conditioned medium from CAFs or NFs was harvested. The conditioned medium was cleared through centrifugation, followed by 1∶1 dilution with defined medium prior to treating the Capan 1 cells; the conditioned medium was freshly transferred without storage.

To obtain CM from QYHJ-treated CAFs, isolated CAFs were plated onto T25 flasks (1 × 10^6^ cells) and cultured in DMEM containing 10% QYHJ-Containing Serum or Control-Containing Serum. Twenty-four hours later, the medium was removed and the cells were washed twice with PBS. Cells were subsequently incubated with 5 ml fresh DMEM medium for an additional 48 hours. The CM was subsequently harvested as described above.

### Enzyme-Linked Immunosorbent (ELISA) assay

The serum CXCL1, 2, and 8 concentrations were measured using an ELISA as previously described [17]. The blood sample was stored at room temperature for 30 min, centrifuged (12000×g) for 15 min, and cryopreserved at -80°C. The concentrations were measured using a sandwich ELISA kit (DuoSet; R&D Systems, Minneapolis, MN, USA). To detect cytokine secretion in the culture medium, the cells were plated onto 6-well plates and treated as described above. After 48 h, the media were collected and stored at −80°C until further use.

### Cell proliferation assay

The cell proliferation assay was performed as previously described [16]. Approximately 5×10^3^ cells in 0.1 ml were plated in duplicate wells of 96-well plates. After overnight incubation, the suspension was removed and changed into different condition media. Subsequently, the indices of cell proliferation were assessed daily using the Cell Counting Kit-8 (CCK-8, Dojindo, Molecular Technologies, Inc, Gaithersburg, MD), and the growth curve was drawn according to the OD values obtain from CCK-8 assay.

### Establishment of xenograft tumor models

Xenograft tumor models were established as previously described [16]. Briefly, Capan1 cells (2×10^6^ in 0.2 ml) in logarithmic phase were injected subcutaneously into the right axilla of nude mice. The length and width of the tumors (in mm) were measured weekly using calipers. The tumor volume was calculated using the formula (a×b^2^)×0.5, where a and b are the long and short dimensions, respectively. The mice were sacrificed when the tumors reached 1.5 cm in diameter. The tumors were removed and weighed. Each group consisted of at least six mice.

### Statistical analysis

The data are expressed as the means ± standard deviation (SD). Statistical analyses were performed using analysis of variance (ANOVA) and Student's t-test. A P-value of <0.05 was considered statistically significant. All statistical analyses were performed using the SPSS 15.0 software package.

## Results

### Generation of cancer-associated fibroblast (CAF) cultures

We extracted fibroblasts from the resected specimens of two pancreatic ductal adenocarcinomas. The tumor masses were dissociated, and various cell types were separated to obtain populations of CAFs. We also isolated a second population of fibroblasts from a noncancerous region of the pancreas at least 2 cm from the outer tumor margin in each of the same two patients. We termed these cells “normal fibroblasts (NFs).” All experiments were performed through comparisons between CAFs and the corresponding NFs, thereby avoiding bias due to interindividual differences. The purity of the cultured fibroblast cells was verified through immunostaining using vimentin and PDGFR-β (mesenchymal cell marker) and E-cadherin and cytokeratin (CK) (epithelial cell marker). In addition, D31 and D2-40 were used to exclude the endothelial origin (Figure 1A and Figure S1). All cell cultures were vimentin and PDGFR-β positive and 91% to 100% E-cadherin, cytokeratin, CD31 and D2-40 negative. Compared with NFs, the established CAFs expressed high levels of alpha smooth muscle actin (α-SMA), a marker of activated fibroblasts, typically expressed in CAF but not normal quiescent fibroblasts. These observations were further confirmed through Western blot analysis (Figure 1B). Taken together, our results indicated that we successfully established paired CAF and NF cultures from human PDAC.

**Figure 1:** Generation and characterization of cancer-associated fibroblast cultures. A. Fibroblasts were extracted from the resected tissues of two pancreatic ductal adenocarcinomas. The purity of the cultured fibroblast cells was verified through immunofluorescence to detect Pan-CK (red), E-cadherin (green), vimentin (red), α-SMA (red), PDGFR-β (red), CD31 (red) and D2-40 (red). The cell nuclei were counterstained with DAPI (blue). Positive control tissues for CD31 and D2-40 immunostaining have been used (Figure S1). B. Western blot analysis confirmed the expression pattern of the markers used in A.

### Pancreatic cancer cells treated with conditioned media from QYHJ-treated CAFs showed reduced invasion

CAFs contribute to the invasive and metastatic process in human pancreatic cancer [5]. In this study, we examined the migration and invasion-inducing effects of CAF on human pancreatic cancer cells using transwell chambers with or without Matrigel coating. The transwell assays demonstrated that the conditioned medium (CM) from control-treated CAFs exhibited an enhanced capacity for inducing pancreatic cancer cell migration and invasion (Figure 2 and Figure S2). Next, we evaluated the effects of QYHJ on CAF-induced cell migration and invasion, the CM from QYHJ or control-treated CAFs were harvested and the effects of this medium on pancreatic cancer cell migration and invasion were also evaluated. We observed that CM from QYHJ-treated CAFs exhibited decreased migration and invasion-promoting capacities compared with that of control-treated CAFs (Figure 2 and Figure S2), these results suggested that QYHJ treatment might suppress pancreatic cancer cell migration and invasion through targeting CAFs.

**Figure 2:** Pancreatic cancer cells treated using conditioned media from QYHJ-treated CAFs showed reduced invasion. The cell migration and invasion capacity of pancreatic cancer cells treated with conditioned media (CM) from NFs, Ctrl-treated CAFs and QYHJ-treated CAFs was compared using transwell chambers with or without Matrigel coating. The numbers of cells that traveled through the membrane were counted in 10 fields under a ×20 objective lens. Original magnification, ×200. The results represent the means ± SD of the values obtained in three independent experiments. Statistical significance was calculated using ANOVA. * *P*<0.05.

### QYHJ inhibits the secretion of CXCL1, 2 and 8 form CAFs

CAFs directly stimulate tumor cell proliferation through various growth factors, hormones and cytokines in a context-dependent manner [5]. We previously showed that CAFs promote the migration and invasion of Capan1 cells in vitro, and this property was inhibited after treated with QYHJ. We next attempted to identify the potential molecules that mediate the correlation between fibroblasts and cancer cells. Previous studies have shown that the members of the CXC chemokine subfamilies, including GRO1 (CXCL1), GRO2 (CXCL2) and IL-8 (CXCL8), are among one of the most highly up-regulated genes identified in CAFs compared with NFs in pancreatic cancer [21]. Therefore, we examined the expression of these factors in CAFs and paired NFs. We observed that CAFs exhibit increased CXCL1, 2 and 8 mRNA and protein expression compared with NFs. In addition, we observed that QYHJ treatment significantly suppressed the expression of CXCL1, 2 and 8 in both CAF cell lines (Figure 3A-B). ELISA assay also confirmed that CAFs treated with QYHJ secreted lower levels of CXCL1, 2 and 8 into the medium (Figure 3C). Thus, these results suggested that QYHJ inhibits the expression of CXCL1, 2 and 8 in CAFs.

**Figure 3:** QYHJ suppressed CXCL production in CAFs. A–B. CAFs were treated with QYHJ-Containing Serum or Control-Containing Serum for 48 h. The cells were then harvested, and the expression of CXCL1, 2 and 8 was evaluated using real-time PCR (A) and western blotting (B). C. The isolated CAFs were plated in T25 flasks (1 × 10^6^ cells) and cultured in DMEM containing 10% QYHJ-Containing Serum or Control-Containing Serum. Twenty-four hours later, the media were removed, and the cells were washed twice with PBS. The cells were subsequently incubated with 5 ml of fresh DMEM medium for an additional 48 hours. The medium was subsequently harvested, and the CXCL1, 2 and 8 concentrations were detected through ELISA. ANOVA was used to determine the statistical significance. * *P*<0.05.

### QYHJ inhibited CAF proliferation in vitro

Previous studies have indicated that the number of CAFs in the stroma is significantly associated with the poor differentiation and prognosis of cancers [22], [23], [24], and reduced CAF numbers were also observed when the tumor was treated[11]. We therefore hypothesized that QYHJ affects CAF proliferation. The in vitro proliferation assay indicated that QYHJ treatment inhibited the proliferation of CAFs in both cell lines (Figure 4), thereby contributing to the suppressed CXC chemokine secretion from CAFs.

**Figure 4:** QYHJ inhibited CAF proliferation in vitro. Approximately 5×10^3^ CAFs in 0.1 ml were plated in duplicate wells of 96-well plates. After overnight incubation, the suspension was removed and transferred to DMEM containing 10% QYHJ-Containing Serum or Control-Containing Serum. The cell proliferation indices were assessed daily using the Cell Counting Kit-8. The results are presented as the means ± SD of values obtained in three independent experiments. *P < 0.05.

### CXCLs increased the migration and invasion of human pancreatic cancer cells

CXC chemokines have been associated with cancer cell invasion in many types of human cancers[25]. As we have observed that CAF exhibited increased CXC chemokines expression and secretion, we confirmed whether the upregulated secretion of CXC chemokines contributes to the enhanced capacity for inducing pancreatic cancer cell migration and invasion. We tested the effects of CXC chemokines on cell migration and invasion using transwell chambers with or without Matrigel coating. The addition of recombinant human CXCL1, 2 and 8 increased both the migration and invasion of Capan 1 cells in the transwell assays. Furthermore, the inhibition of CXC chemokine signaling using receptor antagonists significantly blocked CXC chemokine-induced cell migration and invasion (Figure 5 and Figure S3).

**Figure 5:** CXCLs increased the migration and invasion of human pancreatic cancer cells. Migration and invasion assays were performed on Capan1 cells treated with vehicle, 100/ml CXCL1, 2, and 8, or their antognists 20 µg/ml anti-CXCR1 antibody and 400 nM SB 225002 as indicated, using transwell cell chambers. The number of cells that invaded the membrane was counted in 10 fields under the ×20 objective lens. Original magnification, ×200. The results are presented as the means±SD of values obtained in three independent experiments. The statistical significance was calculated using ANOVA. *P < 0.05.

### QHYJ treatment inhibit tumorigenesis and expression of CXCL1, 2, 8 in vivo

To further confirm the effects of QYHJ on CAF proliferation activity and CXCLs production in vivo, we established mice xenograft models using Canpan1 cells. The mice were randomly divided into QYHJ and control groups, treated with QYHJ (0.2 ml, gavage, daily) or normal saline as a control, respectively. We observed that QYHJ treatment resulted in reduced tumor growth (Figure 6A). Consistent with the results of the in vitro analyses, QYHJ reduced CAF proliferation in tumors (Figure 6B). Moreover, IHC confirmed that tumors treated with QYHJ exhibited the reduced expression of CXCL1, 2, and 8 (Figure 6D). Therefore, our results suggested that QHYJ treatment inhibited CAF proliferation and the expression of CXCL1, 2, and 8, potentially reflecting the anti-cancer effects of QHYJ in pancreatic cancer.

**Figure 6:** QHYJ treatment inhibited tumor growth and the expression of CXCL1, 2, and 8 in vivo. A. Effect of QYHJ on tumor growth in a subcutaneously transplanted tumor model. Capan1 cells (2 × 10^6^cells in 200 ml) were injected subcutaneously into the right axilla of each BALB/c-nu/nu nude mouse. The next day, the mice were orally treated with or without QYHJ. The mean tumor volumes of vehicle-treated (saline water) and QYHJ-treated tumors were measured. The mean ±standard deviation was determined in each treatment group. The tumor growth curves are shown in the upper panel, and photographs of subcutaneously transplanted tumors from both groups are shown in the lower panel. Student's t-test was used to determine the statistical significance. *P < .05 compared with the QYHJ-treated group. B. IHC staining for vimentin and α-SMA on sections of tumors to evaluate CAF proliferative activities. A arrow indicates fibroblast and arrowhead indicates pancreatic cancer cell. Original magnification, 200×. CAF proliferative activities (right) were quantitatively evaluated after calculating the ratio of the vimentin or α-SMA antibody-positive staining area to the total area in each field, and the mean value from ten fields under 200× microscopy are indicated. *P < 0.05. C. IHC staining using anti-CXCL1, 2, and 8 antibodies was performed using sections of transplanted tumors. Original magnification, ×200. The positive rates of CXCL1, 2, and 8 in tumors are shown on the right. Student's t-test was used to determine the statistical significance. *P < 0.05.

## Discussion

In this study we showed that the QYHJ inhibits pancreatic cancer cell invasion and metastasis by targeting CAFs, particularly the production of CXCL1, 2, and 8. These findings further confirmed our previous speculation that cells in the tumor microenvironment might serve as pivotal targets for Chinese herbal medicine[11].

Traditional Chinese medicine (TCM) is based on a unique theory formed in lone-term practical experience. For the last thousand years, TCM has been widely practiced in China, and more than 90% of modern Chinese cancer patients have received TCM therapy during treatment [26]. Recently, TCM has been used abroad and is well accepted in many countries, particularly for the treatment of oncology [27]. TCM is based on the concept of holism, considering the interrelationship of the human body and the surrounding environment on the macro level. At the microscopic scale, we consider the holistic relationship between cancer cells and the microenvironment. Indeed, recent studies have confirmed that tumor cells do not act in isolation, but rather subsist in a rich microenvironment provided by resident fibroblasts, inflammatory cells, endothelial cells, pericytes, leukocytes, and the extracellular matrix [28]. As the cancer progresses, the surrounding microenvironment is activated, coevolving through continuous paracrine communication, to support carcinogenesis [29]. Pancreatic cancer is characterized by an extensive stromal response called desmoplasia [7]. CAFs are the primary cell type in the tumor stroma, and the importance of a role for CAFs in tumor progression is well accepted [5]. Therefore, as cancer is no longer considered a discrete entity defined only through the traits of cancer cells within the tumor, eventually affecting the entire organism, TCM offers a holistic approach to regulate the integrity of all body functions and the interaction between the humans and the surrounding environment. Targeting the tumor microenvironment might represent a potential therapeutic approach for pancreatic cancer treatment.

QYHJ is a seven-herb Chinese formula used in the treatment of pancreatic cancer in China. We previously showed that QYHJ inhibits both tumor growth and metastasis in nude mice with pancreatic cancer models [12], [13]. The combination of QYHJ treatment with conventional Western medicine prolongs survival in patients with pancreatic cancer liver metastases [14].The exact mechanism underlying the effects of QYHJ in pancreatic cancer treatment remains unclear. Recent studies have indicated that QYHJ treatments dramatically alter the tumor microenvironment, observed through decreased CAF proliferation [11]. Therefore, in this study, we further evaluated the effects of QYHJ on CAF proliferation and the production of CAF-derived chemokines. We observed that QYHJ inhibited CAF proliferation both in vitro and in vivo. In addition, the inhibition of CXCL production through QYHJ treatment resulted in the reduced invasion of pancreatic cancer cells. Thus, this study was the first to identify a new target of pancreatic cancer cells using Chinese herbal medicine.

CXCL1, 2, and 8, produced primarily by mononuclear cells, macrophages and a smaller percentage of fibroblasts, endothelial cells, T and B lymphocytes, chondrocytes and amnion cells, are pleiotropic cytokines that induce tumor formation, promote tumor proliferation and facilitate tumor metastasis [30], [31]. Increasing evidence has shown that CXCL1, 2, and 8 are frequently elevated in many types of human cancers [30], [32], [33], [34], including pancreatic cancer [31]. In addition, therapies targeting CXCL1, 2, and 8 in the treatment of cancers have been reported [30], [35], [36], and the down-regulation of CXCL1, 2, and 8 inhibited the invasion of tumor cells [32] [35]. Using in vitro function assays, we demonstrated that CAFs exhibit increased CXCL1, 2 and 8 expression in pancreatic cancer, contributing to the enhanced invasion-promoting capacity of these cells. Therefore, targeting CXC chemokine signaling between CAF and cancer cells through pharmacological inhibition might provide a promising therapy for pancreatic cancer. The results obtained in the present study showed that Chinese herbal medicine QYHJ could significant suppress the production of CAF-derived CXCL1, 2 and 8, thereby preventing pancreatic cancer cell invasion.

Thus, in this study, we have demonstrated that CAFs exhibited an enhanced capacity for inducing pancreatic cancer cell migration and invasion compared with NFs, while QYHJ-treated CAFs exhibited decreased migration and invasion-promoting capacities in vitro. In addition, we showed that QYHJ significantly suppressed CAF proliferation activities and the production of CAF-derived CXCL1, 2 and 8. Taken together, these results suggested that suppressing the tumor-promoting capacity of CAFs through Chinese herbal medicine attenuates pancreatic cancer cell invasion.

## Supporting Information

Figure S1 **Positive control for CD31 and D2-40 immunostaining.** (A) The positive control for CD31 is vascular endothelium in pancreas. (B) The positive control for D2-40 is lymphatic endothelium in lymph node.
(TIF)

Figure S2 **Pancreatic cancer cells BxPC3 treated using conditioned media from QYHJ-treated CAFs showed reduced invasion.** The cell migration and invasion capacity of pancreatic cancer cells BxPC3 treated with conditioned media (CM) from NFs, Ctrl-treated CAFs and QYHJ-treated CAFs was compared using transwell chambers with or without Matrigel coating. The numbers of cells that traveled through the membrane were counted in 10 fields under a ×20 objective lens. Original magnification, ×200. The results represent the means ± SD of the values obtained in three independent experiments. Statistical significance was calculated using ANOVA. * *P*<0.05.
(TIF)

Figure S3 **CXCLs increased the migration and invasion of human pancreatic cancer cells BxPC3.** Migration and invasion assays were performed on BxPC3 cells treated with vehicle, 100 ng/ml CXCL1, 2, and 8, or their antognists 20 µg/ml anti-CXCR1 antibody and 400 nM SB 225002 as indicated, using transwell cell chambers. The number of cells that invaded the membrane was counted in 10 fields under the ×20 objective lens. Original magnification, ×200. The results are presented as the means±SD of values obtained in three independent experiments. The statistical significance was calculated using ANOVA. *P < 0.05.
(TIF)
